# Identification and Prediction of Chronic Diseases Using Machine Learning Approach

**DOI:** 10.1155/2022/2826127

**Published:** 2022-02-25

**Authors:** Rayan Alanazi

**Affiliations:** Department of Computer Science, College of Science and Arts in Qurayyat, Jouf University, Sakakah, Saudi Arabia

## Abstract

Nowadays, humans face various diseases due to the current environmental condition and their living habits. The identification and prediction of such diseases at their earlier stages are much important, so as to prevent the extremity of it. It is difficult for doctors to manually identify the diseases accurately most of the time. The goal of this paper is to identify and predict the patients with more common chronic illnesses. This could be achieved by using a cutting-edge machine learning technique to ensure that this categorization reliably identifies persons with chronic diseases. The prediction of diseases is also a challenging task. Hence, data mining plays a critical role in disease prediction. The proposed system offers a broad disease prognosis based on patient's symptoms by using the machine learning algorithms such as convolutional neural network (CNN) for automatic feature extraction and disease prediction and K-nearest neighbor (KNN) for distance calculation to find the exact match in the data set and the final disease prediction outcome. A collection of disease symptoms has been performed for the preparation of the data set along with the person's living habits, and details related to doctor consultations are taken into account in this general disease prediction. Finally, a comparative study of the proposed system with various algorithms such as Naïve Bayes, decision tree, and logistic regression has been demonstrated in this paper.

## 1. Introduction

All over the world, chronic diseases are a critical issue in the healthcare domain. According to the medical statement, due to chronic diseases, the death rate of humans increases. The treatments given for this disease consume over 70% of the patient's income. Hence, it is highly essential to minimize the patient's risk factor that leads to death. The advancement in medical research makes health-related data collection easier [1, 2]. The healthcare data includes the demographics, medical analysis reports, and the history of disease of the patient. The diseases caused could be varied based on the regions and the living habitats in that region. Hence, along with the disease data, the environmental condition and the living habitat of the patient should also be recorded in the data set.

In recent years, the healthcare domain is evolving more due to the integration of information technology (IT) in it. The intention to integrate IT in healthcare is to make the life of an individual more affordable with comfort as smartphones made one's life easier [3]. This could be possible by making healthcare to be intelligent, for instance, the invention of the smart ambulance, smart hospital facilities, and so on, which helps the patients and doctors in several ways [4]. The research on a specified region for patients affected by chronic diseases every year had been held and found that the difference between the patients in genderwise is very small, and it is found that the large number of patients were admitted in the year 2014 for treating chronic diseases. The use of structured and unstructured data provides highly accurate results instead of using only structured data. Since the unstructured data includes the doctor's records on the patients related to diseases and the patient's symptoms and grievances faced by them, explained by themselves, which is an added advantage when used along with the structured data that consists of the patient demographics, disease details, living habitats, and laboratory test results [5, 6]. It is difficult to diagnose rare diseases. Hence, the use of self-reported behavioral data helps differentiate the individuals with rare diseases from the ones with common chronic diseases. By using machine learning approaches along with questionnaires, it is believed that the identification of rare diseases is highly possible [7].

In the last decade, some innovative technologies had been introduced to rapidly collect the data such as MRI (magnetic resonant imaging) readouts, ultrasonography, social media gained data, and electronically gained activity, behavioral, and clinical data. These big data sets of healthcare are high-dimensional, which means the number of features recorder per observation might be greater than the total observations. They are noisy, sparse, cross-sectional, and lacks statistical power. By applying machine learning techniques, the issues in the high-dimensional data sets can be overcome [8]. Machine learning contributes more in several domains. Many of the complex models make use of exiting larger training data, simultaneously at the edge of a major shift in healthcare epidemiology [9]. These data can enhance the knowledge gain in the risk factors of diseases to reduce healthcare-associated infections, improve patient risk stratification, and find the way of transmitting the infectious diseases [10]. Machine learning can facilitate the analysis of laboratory results and other details of patients for the early detection of diseases. The low-level data could be converted to high-level knowledge via knowledge discovery in the database so as to gain knowledge about the disease patterns to support early detection [11]. The data collected for creating a data set should be preprocessed for its missing values, and then only the important features needed for accurate disease prediction are selected so as to enhance the prediction accuracy and minimizing the time taken for model training [12].

In the era of the Internet and technologies, people are not concerned about their health and lives. As everyone is interested in surfing and social media activities, they ignore visiting hospitals for their health checkup. By taking this activity as an advantage, a machine learning model that takes the symptoms given as input and predicts the possibility and risk of the disease affected or the development of such diseases in an individual should be developed [13, 14]. The more common chronic diseases are diabetes, cardiovascular diseases, cancer, strokes, hepatitis C, and arthritis. As these diseases persist for a long time and have a high mortality rate, the diagnosis of such diseases is highly important in the healthcare domain. Foreseeing the disease can help take preventive actions and avoid getting affected by it, and early detection of it can help provide better treatment [15]. There are various techniques in machine learning such as supervised, semisupervised, unsupervised, reinforcement, evolutionary, and deep learning. The problem is associated with the processing of extracted features from real data and structured as vectors [16]. The processing quality is based on the proper combination of those vectors. But, most of the times, the high dimensionality of the vectors or the discrepancies in the data makes a big issue. Hence, it is important to reduce the dimensionality of the data set even if it leads to a little loss of details to make the data set a highly compatible dimension. This reduction in the dimensionality of the data set improves the model performance [17].

The system of chronic diseases management is essential for those affected by such diseases and in need of proper medical assessment and treatment information [18]. Also, this system can be useful for individuals who are in need of self-care to improve their health condition, since it is proved that self-management is the primary care of those with chronic diseases, and it is considered as the unavoidable part of treatment. With the use of mobile applications, the health information of patients can be recorded, and they serve as a better tool to enable self-management [19]. To effectively predict a disease, information such as narration about the symptoms felt by the patients, details of consultation with medical practitioners, lab examination results, and computed tomography and X-ray images [20]. Little research is performed in identifying the accuracy and predictive power for developing a machine learning model with only information from lab examination results for the diagnosis of diseases. And, for performance enhancement, ensemble machine learning and deep learning model can be used [21, 22]. In the healthcare domain, artificial intelligence (AI) plays a major role in automating the roles involved in disease diagnosis and treatment suggestions and also schedules perfect timing by the medical practitioners to perform various obligations that cannot be automated [23].

The major objective of the proposed system is to identify and predict chronic disease in an individual using a machine learning approach [24, 25]. The data set comprises both the structured data that includes the patient's age, gender, height, weight, and so on, excluding the patient's personal information such as name and ID, and the unstructured data that includes the patient's symptoms, information related to consultation about the disease with the doctors, and the living habits of that individual [26]. These data are preprocessed for finding the missing values. They are then reconstructed to increase the quality of the model, thereby increasing the prediction accuracy. For prediction, the machine learning algorithms such as CNN and KNN are used [27, 28]. This paper is organized as the details of the related works carried out while doing the research are given in Section 2, the preliminaries of the algorithms used in given in Section 3, the description of the proposed methodology in Section 4, the result and discussion part are given in Section 5 followed by the conclusion in Section 6, and finally, a list of references used in this study has been given.

## 2. Related Work

This section describes the related works that are performed in developing the proposed model for predicting chronic diseases. The following are the discussions made by reviewing the existing literature that helps develop the proposed system efficiently and effectively.

The objective variable of the study in [29] is the resource consumption such as medical and long-term care expenses and a predictive model for medical care using a random forest machine learning algorithm [30]. This method uses data of more than 100 pieces that includes preventive activities, clinical tests, and medical practices. This model uses mean decrease Gini for classification and for regression mean square error (MSE) is used [31, 32]. The training model uses a grid search for hyperparameter tuning and is validated using *K*-fold cross-validation. Along with the objective variable, exploratory variables such as age, gender, and analysis period are also included, since the aim of this paper is proper management of the budget for medical care [33]. A review that highlights the applications of machine learning techniques in various medical practices such as predicting, diagnosing, and prognosis of diseases such as multiple sclerosis, autoimmune chronic kidney disease, autoimmune rheumatic disease, and inflammatory bowel disease and for the selection of treatments and stratification of patients; drug development; drug repurposing; target interpretation; and validation has been given in [34, 35]. This paper also provides a detailed description of the challenges faced by the machine learning approaches such as the need for quality data in preparation of robust models, external model validation using the independent data set, difficulties faced during implementation of a model, and ethical concerns. A predictive model for chronic kidney disease is explained in [36, 37]. This model is developed using four machine learning approaches such as support vector machine (SVM), logistic regression (LR), decision tree (DT), and KNN for classification purposes. The data set used in this paper is the Indian chronic kidney disease (CKD) that consists of 400 occurrences, 24 features, and 2 classes obtained from the UCI machine learning repository. The developed model is evaluated using a 5-fold cross-validation process, and the experiment is conducted on the Weka data mining tool and MATLAB and finally concluded that the SVM classifier attains higher accuracy when compared to the others.

A system that can predict multiple diseases with the help of various machine learning algorithms such as Naïve Bayes, KNN, DT, random forest, and SVM algorithms has been described in [38] to bridge the gap among the patients and the doctors to achieve their own goals. The existing approaches in the field of automatic disease prediction lack the patient's trust in the model's prediction and also reduce the need for doctors, which makes the doctors get panic about their livelihood. But this method integrates a module for doctor recommendation that solves both the issues by making sure the patient to trust due to the intervention of doctors and also improves the business of doctors. A model called PARAMO, which is a platform of a parallel predictive model that uses electronic health records (EHR) for healthcare analysis, has been implemented in [39]. This method comprises three phases, namely, the generation of the dependency graph, which removes redundancy and identifies dependency; then execution engine for dependency graph, which includes prioritizing, scheduling, and parallel execution; and finally the parallelization infrastructure. The PARAMO model is tested with three sets of real data, that is, small, medium, and large data sets that includes the medications, diagnosis data, and lab records, obtained from EHR that ranges from 5,000 to around 300,000 patients. In addition to this, the small and large sets include the procedure data, and the medium set includes the symptoms of heart failure that are taken from medical records [40]. An efficient recommendation system for chronic disease diagnosis has been demonstrated in [41]. This method uses a data mining approach. The data set used in this system includes medical data and two-dimensional data. The medical data include the data obtained from sensors or medical data entries, and the two-dimensional data include the external user and the item features. For enhancing the accuracy of prediction, the decision tree approach, which is a highly prevalent data mining approach, is used for classification. Various decision tree classifiers such as random forest, REP tree, decision stump, and J48 are involved in the creation of this predictive model. This model is tested with randomly selected 20 samples and found that the RF outperforms the other three algorithms.

Prediction of 3 types of immune diseases such as allergy, infectious, and autoimmune diseases using decision tree, maximum margin learning, and instance-based learning, respectively, has been given in [42]. The correlation between the classification of immunogens and its physicochemical properties is one of the purposes of this study. The immunogen data such as the stats of diseases, responses from B-cell, discontinuous epitope location, host, source organisms, and so on are collected from Immune Epitope Database (IEDB) and analyzed its 6 physicochemical properties such as PSSM (position-specific scoring matrix) information per position, hydrophilic scale, flexibility, antigenic propensity, hydropathy index, and side chain polarity. This system is tested using a method called leave-one-out cross-validation for the performance of prediction outcomes with parameters such as accuracy and F-score. A risk prediction model for predicting disease risks using a random forest machine learning approach from highly imbalance data has been described in [43]. The data set used in this approach is the Nationwide Inpatient Sample (NIS), which includes 8 million records of hospital stays with 126 clinical as well as nonclinical data. The nonclinical data comprises patient's demographics, hospital location, date and year of admission, pin code, treatment/diagnosis cost, and duration of stay in a hospital ward. The clinical data comprises the treatment procedures, its categories, diagnosis categories, and its codes. Each record has a vector containing 15 diagnosis codes characterized by International Classification of Diseases, 9^th^ Revision, Clinical Modification (ICD-9-CM). As the unbalance data produces undesirable results, a repeated random sampling method is employed to solve this issue. The developed model is evaluated using SVM, RF ensemble learning, bagging, and boosting algorithms. The study [44] demonstrates a novel adaptive probabilistic divergence-based feature selection algorithm to predict chronic kidney disease in its earlier stage. This algorithm is based on statistical and divergence information theory. For classification, the hyperparameterized logistic regression model is used in this study. The data set used in this approach is obtained from various hospitals and laboratories with information of 630 patients with 52 attributes, and this data set is given to the physician for verification of its correctness. The model developed is evaluated using the data sets of diabetes, heart, and kidney diseases, and the performance evaluation metrics followed in this study is the precision, recall, F1-score, and ROC (receiver operating characteristics) curve.

A system that enhances the risk prediction of a patient's health condition using a deep learning approach on big data and a revised fusion node model has been demonstrated in [45]. This deep learning model for extracting the data and logical inference is made of the combination of complex machine learning algorithm such as Bayesian fusion and neural networks. The architecture of this system consists of five layers, namely, the data layer that is responsible for data collection, data aggregation layer for data acquisition from several data sources and desired format changing, analytics layer to do proper analytics on the data aggregated, information exploration layer to create the output that makes the results of analytics understandable for users, and big data governance layer that is responsible for managing the above layers. Also, in this paper, the application of MapReduce is discussed for optimizing the analytics efficiency and also inspires the design of SOA (service-oriented architecture) for making the external systems easily access the results from analytics. A machine learning model of disease prediction cost has been implemented in [46] that uses big data, which includes structured and unstructured data for preparing the data set and the developed model is made available at affordable. The prediction algorithm used in this method is the decision tree algorithm and the MapReduce algorithm is applied for enhancing the efficiency of the operation. The advantages of this model are reduction in retrieval time of queries, improved accuracy. A method of predicting the risk of chronic kidney disease using zub machine learning approaches has been described in [47, 48]. Two types of data sets are used in this method. One is from UCI with 400 instances and 35 features, and the other is a real-time data set obtained from Khulna City Medical College with 55 instances and 25 features. Data processing is done using Pandas and Numpy libraries, and the missing data are handled using median filtering. Feature extraction is performed using the Chi-square test. Model evaluation is performed using 10-fold cross-validation. Artificial neural network (ANN) and random forest algorithms are used for disease classification. This method is believed that it can predict the risk of chronic kidney disease in its earlier stage [49–52].

## 3. Preliminaries

### 3.1. Chronic Disease

According to US National Center for Health Statistics, chronic diseases are diseases that last for a long period of time, that is, more than three months. These diseases are neither treated by medicines nor prevented by vaccines. The major cause of chronic diseases is the use of tobacco, unhealthy food habits, and lack of physical activity. Also, this disease can commonly be caused due to ageing. Chronic diseases include cardiovascular disease, cancer, arthritis, diabetes, obesity, epilepsy and seizures, and problems in oral health [35].

Cardiovascular disease includes heart disease and stroke, which highly lead to death. This disease is caused due to the use of tobacco, intake of nutritionless food, and lack of physical activity. When these activities are changed by the patient, they might have the chance to reduce the impact on controlling and preventing cardiovascular disease.

Next to cardiovascular disease, cancer such as colon cancer and breast cancer is considered the deadliest disease. It can be controlled only by prevention, early detection, and proper medical support. Minimizing the prevalence of environmental and behavioral factors that causes cancer reduces the chance risk of causing it.

The chronic disease such as arthritis causes inflammation in the joints, causes pain, and stiffness that increases due to ageing. There is an availability of cost-effective methods for reducing the effects caused by arthritis but are not used much. The effects of arthritis can be reduced by following moderate exercises regularly.

Diabetes is a serious and high-money-consuming disease. The impact of diabetes can be reduced by self-care and early detection of the disease [53]. Around 7 million people over the age of 65 or above are affected by this disease particularly type 2 diabetes.

Since 1980, obesity is more common in adults for all age groups. The one who is overweight or obese can develop the risk of getting high blood pressure (BP), heart diseases, diabetes, and arthritis. Obesity can also cause some types of cancers.

Epilepsy and seizures are highly costly in treatment [54]. This disease is common among all age groups, especially in young and elders.

Oral health problems are a crucial issue that attains special attention in the health of older people. This is a serious issue, since it affects the normal day-to-day actions of a person such as speak, chew, swallow, and maintain a nutritional food plan.

### 3.2. Convolutional Neural Network (CNN)

The ConvNet or CNN is an algorithm of deep learning that fetches the input and assigns the bias and weights to its several aspects and then distinguishes one from the other [55] as shown in Algorithm 1. The major reason for using CNN is that it requires only few efforts in preprocessing the data when compared with other algorithms, since the CNN can learn to optimize the filters through automate learning [56]. The output layer of CNN can be calculated using the following expression:

(1) $$\begin{array}{c} \text{size of output layer}=\text{input size}-\left(\text{filter size}-1\right). \end{array}$$

### 3.3. K-Nearest Neighbor (KNN)

KNN is a supervised machine learning algorithm, which analyzes the similarities between the new data and the existing data and adds the new data into the category that is highly similar to the available categories [57] as shown in Algorithm 2. The KNN can be used in classification as well as regression tasks, but it is most commonly used in classification. This algorithm is also called the lazy learner algorithm; since it will not learn instantly from the training data, it stores the data set and does its action during the classification process. The calculation of Euclidean distance is expressed mathematically as follows:

(2) $$\begin{array}{c} x^{2}=c-a^{2}+d-b^{2}. \end{array}$$

## 4. Proposed Methodology

In this section, a detailed description of the data set creation, model preparation, and disease prediction has been given. The first action is data collection. Our proposed system collects structured and unstructured data obtained from various sources. After data collection, they are subjected to preprocessing and are split into cleaning and test data sets. Then the training data set is trained with the machine learning algorithms such as CNN and KNN to a number of epochs for improving the accuracy of the prediction results. After multiple epochs, once the desired target is achieved, the developed model is ready for testing.

At this step, the model is tested with the test data set to verify the model performance with brand-new data that were not used for training. If the model attains the desired accuracy in test data, then the proposed model is ready for deployment as shown in Figure 1.

### 4.1. Data Collection

The real-life data that includes structured data such as patient basic information including demographics, living habitat, and lab test results and the unstructured data such as the symptoms of the disease faced by the patient and their consultation with the doctor. The data set excludes the patient's personal details such as name, ID, and location so as to preserve their privacy.

### 4.2. Preprocecssing

The collected data are preprocessed for the availability of missing values in most of the structured data. Hence, it is essential to fill out the missed data or remove or modify them to enhance the quality of the data set. The preprocessing step also eliminates the commas, punctuations, and white spaces. Once the preprocessing of data has been completed, it is then subjected to feature extraction followed by disease prediction.

### 4.3. Model Description

As discussed above, the data set consists of both structured and unstructured data. The structured data comprises patient demographics and the data related to the cause for the disease such as age, gender height, weight, and so on, patient's living habitat, laboratory test results, and the disease that they are affected in tabular format. The unstructured data comprises patient's disease symptoms and the information about the interrogation with doctors in text format. The unstructured data is an added advantage of the prediction task to get a more accurate results. The data set is split into 80% for training and 20% for testing.

### 4.4. Disease Prediction Using CNN

The proposed system uses the CNN algorithm in the prediction of chronic disease. At first, the data set is converted into vector form, followed by word embedding to adopt zero values for filling the data. It is then given to the convolution layer.

The pooling layer takes the input from the convolution layer and follows the max pooling operation. The output of max pooling is given to the fully connected layer, and then finally, the output layer provides the classification results.  Figure 2 shows the block diagram of the convolutional neural network.

### 4.5. Distance Calculation Using KNN

In *K*-Nearest Neighbor (KNN), the value of *K* is known, and the features that are similar to the *K* value are called the nearest neighbor. The nearest neighbor to the known *K* value is chosen, and the nearest distance between them is calculated. The feature with less distance value is considered to be the exact match, which is the final disease prediction output. In the proposed system, Euclidean distance is used, since the result obtained by it is better when compared to other distance calculation methods. It is a nonparametric algorithm since it will not take decisions on original data. In KNN, the training input data are located in *X* and *Y* axes, and the test data are located in the plots of *X* and *Y* axes. Then, the plots of test data with less distance are chosen and are considered as the desired target. It is important to choose the value of the nearest *K* point should be always odd.

The calculation of Euclidean distance can be performed by using the following formula and is represented in Figure 3:

(3) $$\begin{array}{c} D=\sqrt{{\left(X_{1}-Y_{1}\right)}^{2}+{\left(X_{2}-Y_{2}\right)}^{2}+\cdots +{\left(X_{n}-Y_{n}\right)}^{2}}. \end{array}$$

## 5. Performance Evaluation

For evaluating the proposed disease prediction model, four performance evaluation metrics are used. The confusion matrix consists of the true positives (TP), which is the correct prediction of the target as a patient with chronic disease; the true negatives (TN), which is the correct prediction of the persons without diseases; false positives (FP), which is the incorrect prediction of the healthy person as a diseased person, and false negatives (FN), which is the incorrect prediction of the target as healthy persons. The following is the description of the four performance evaluation parameters.

### 5.1. Accuracy

The classification accuracy is described as the ratio of correct predicted values to the total predicted values and is depicted mathematically as follows:

(4) $$\begin{array}{c} \text{Accuracy}=\frac{\text{TP}+\text{TN}}{\text{TP}+\text{TN}+\text{FP}+\text{FN}}*100. \end{array}$$

### 5.2. Precision

The precision or positive predictive value (PPV) is described as the ratio of correct prediction to the total correct values including the true and false predictions and is depicted mathematically as follows:

(5) $$\begin{array}{c} \text{Precision}=\frac{\text{TP}}{\text{TP}+\text{FP}}. \end{array}$$

### 5.3. Recall

The recall or sensitivity or true positive rate (TPR) is described as the ratio of correct predicted values to the sum of correct positive predictions and the incorrect negative predicted values and is depicted mathematically as follows:

(6) $$\begin{array}{c} \text{Recall}=\frac{\text{TP}}{\text{TP}+\text{FN}}. \end{array}$$

### 5.4. F1-Score

The F-measure (*F*_*β*_) is described as the weighted average of the values obtained from the calculation of precision and recall parameters. Whenever the distribution of class is not even, then the value of *F*_1_ − Score is highly important than the accuracy value. And whenever the values of false positives and negatives are dissimilar, the value of *F*_1_ − Score is highly suitable. The *F*_1_ − Score is depicted mathematically as follows:

(7) $$\begin{array}{c} F_{\beta }=\frac{\left(1+\beta^{2}\right)\left(\text{Precision}*\text{Recall}\right)}{\left(\beta^{2}*\left(\text{Precision}+\text{Recall}\right)\right)}. \end{array}$$

By simplifying using *β*=1,

(8) $$\begin{array}{c} F_{1}-\text{Score}=2*\frac{\text{Precision}*\text{Recall}}{\text{Precision}+\text{Recall}}. \end{array}$$

The obtained values of precision, recall, and F1-score of the proposed CNN and KNN model is compared with the values of the performance metrics of Naïve Bayes, decision tree, and logistic regression algorithms, and the results are tabulated in Table 1.

The accuracy is the important parameter since the prediction result is the important factor for the patient, and if it is wrong, then it will be a detriment to them. The other parameters such as precision, recall, and F1-score are for the evaluation of the model performance as shown in Table 1.

Figure 4 shows the graphical representation of the comparison results of accuracies of the proposed and other algorithms. This graph illustrates the variations in the prediction accuracies of the four algorithms such as the Naïve Bayes, decision tree, logistic regression, and the proposed CNN and KNN algorithms as 52%, 62%, 86%, and 96%, respectively. This shows that the proposed system achieves the highest accuracy of 96% when compared to the other machine learning algorithms.

Figure 5 shows the graphical representation of the comparison precision, recall, and F1-score values of the proposed and other algorithms. This graph illustrates the variations in the three performance evaluation parameters of the four algorithms such as the Naïve Bayes, decision tree, logistic regression, and the proposed CNN and KNN algorithms as 52%, 64%, 84%, and 93%, respectively, for precision; 80%, 605, 88%, and 99%, respectively, for recall; and 65%, 62%, 82%, and 97%, respectively, for F1-score. These results shows that the prosed model developed using CNN and KNN algorithm is considered to be the best of the remaining three algorithms with 93%, 99%, and 97% for precision, recall, and F1-score, respectively, which is higher when compared to the others.

## 6. Conclusion

This paper proposed a method of identification and prediction of the presence of chronic disease in an individual using the machine learning algorithms such as CNN and KNN. The advantage of the proposed system is the use of both structured and unstructured data from real life for data set preparation, which lacks in many of the existing approaches. In this paper, the performance of the proposed model is compared with other algorithms such as Naïve Bayes, decision tree, and logistic regression algorithms. The results show that the proposed system provides an accuracy of 95% that is higher than that of the other two algorithms. It is highly believed that the proposed system can reduce the risk of chronic diseases by diagnosing them earlier and also reduces the cost for diagnosis, treatment, and doctor consultation.

## Figures and Tables

**Figure 1:** Architecture of proposed disease and risk prediction system.

**Figure 2:** Block diagram of convolutional neural network.

**Figure 3:** Calculation of Euclidean distance.

**Figure 4:** Comparison of accuracies of proposed and other algorithms.

**Figure 5:** Comparison of other performance evaluation metrics of proposed and other algorithms.

**Algorithm 1:** Convolutional neural network algorithm.

**Algorithm 2:** K-nearest neighbor algorithm.

**Table 1:** Performance evaluation comparison.

	Accuracy (%)	Precision (%)	Recall (%)	F1-score (%)
Naïve Bayes	52	52	80	65
Decision tree	62	64	60	62
Logistic regression	86	84	88	82
CNN and KNN	96	93	99	97

## Data Availability

The data used to support the findings of this study are included within the article.
